# Human Centered Decision-Making for COVID-19 Testing Center Location Selection: Tamil Nadu—A Case Study

**DOI:** 10.1155/2022/2048294

**Published:** 2022-03-10

**Authors:** S. Saroja, R. Madavan, S. Haseena, M. Blessa Binolin Pepsi, Alagar Karthick, V. Mohanavel, M. Muhibbullah

**Affiliations:** ^1^Department of Information Technology, Mepco Schlenk Engineering College, Sivakasi, 626005 Tamil Nadu, India; ^2^Department of Electrical and Electronics Engineering, PSR Engineering College, Sivakasi, 626140 Tamil Nadu, India; ^3^Renewable Energy Lab, Department of Electrical and Electronics Engineering, KPR Institute of Engineering and Technology, Coimbatore, 641407 Tamil Nadu, India; ^4^Centre for Materials Engineering and Regenerative Medicine, Bharath Institute of Higher Education and Research, Chennai, 600073 Tamil Nadu, India; ^5^Department of Electrical and Electronic Engineering, Bangladesh University, Dhaka 1207, Bangladesh

## Abstract

This paper proposes a blend of three techniques to select COVID-19 testing centers. The objective of the paper is to identify a suitable location to establish new COVID-19 testing centers. Establishment of the testing center in the needy locations will be beneficial to both public and government officials. Selection of the wrong location may lead to lose both health and wealth. In this paper, location selection is modelled as a decision-making problem. The paper uses fuzzy analytic hierarchy process (AHP) technique to generate the criteria weights, monkey search algorithm to optimize the weights, and Technique for Order of Preference by Similarity to Ideal Solution (TOPSIS) method to rank the different locations. To illustrate the applicability of the proposed technique, a state named Tamil Nadu, located in India, is taken for a case study. The proposed structured algorithmic steps were applied for the input data obtained from the government of India website, and the results were analyzed and validated using the government of India website. The ranks assigned by the proposed technique to different locations are in aligning with the number of patients and death rate.

## 1. Introduction

The unique coronavirus disease-caused pandemic, which first surfaced in December 2019 and causes a contagious severe acute respiratory sickness in people, is sweeping the globe and causing great alarm [1]. The World Health Organization (WHO) has dubbed the virus coronavirus disease 2019 (COVID-19) and has asked all nations to work together immediately and decisively to contain it. It affects the human respiratory system and is very similar to the influenza virus. Fever, cough, cold, nausea, exhaustion, breathing problems, and other serious symptoms are caused by it [2]. It is a global health epidemic that is affecting millions of people all over the world and spreading like wildfire. Many limitations have been placed on travel, meetings, and gatherings in public locations in order to prevent the virus from spreading. As asymptomatic transmission has made limiting the spread more difficult, social isolation and testing may be used to combat the pandemic.

Because fever is one of the symptoms of coronavirus, temperature screening alone was initially utilized to diagnose COVID-19. However, because infected people could still be in the incubation period and not display any symptoms, this method failed to provide accurate results. Reverse transcription-polymerase chain reaction (RT-PCR) assays are the most accurate way to determine the pathogen that causes COVID-19. RT-PCR assays are utilized to diagnose COVID-19 in India and around the world. Nasal and throat swabs are utilized to determine the virus presence in the human body. This test detects viral RNA in the bloodstream. Other testing methods, such as rapid antibody tests, rapid antigen tests, and TrueNat tests, are also used in India. According to the Ministry of Health and Family Welfare [3], the total number of confirmed cases in India approached twenty-five lakhs on August 17, 2020, with over 50,000 fatalities. The overall number of COVID-19 tests performed each day in India has increased from a few thousand in March to nearly ten thousand in August. If someone is suspected of having COVID-19, they should be tested anyway. The government provides this test for free, but private hospitals charge different fees.

As the number of coronavirus-infected patients in India grows, the Union Health Ministry is expanding the number of COVID-19 testing labs to 1504, with 978 government labs and 526 private labs doing RT-PCR, TrueNat, and CBNAAT-based COVID-19 tests [4]. The easiest method to keep the spread under control is to test samples early on. The proposed study will determine the location of a new testing center that the government plans to deploy based on a variety of criteria and alternatives.

Researchers in [5] developed software called VECTOR to process the lung sounds for identifying the presence of interstitial pneumonia. Machine learning techniques [6, 7] and deep learning techniques [8, 9] are also employed for the early diagnosis of COVID. Natural products based on flavonoids for COVID are suggested [10]. The proposed work applies metaheuristic techniques to optimize the generated weights. In recent days, researchers are applying a wide variety of metaheuristic algorithms [11–18] like the monarch butterfly optimization, slime mould algorithm, moth search algorithm, and colony predation algorithm quite often rather than the exact method due to the simplicity and robustness of the obtained results. Exact methods incur high computation times, whereas metaheuristic techniques will find optimal solutions at reasonable computation times. The monkey search algorithm (MSA) is introduced in [19], and it is applied to solve optimization problems like scheduling, clustering, and so on [20–23]. It is deployed in the proposed work to optimize the weight generated from fuzzy AHP. It is based on the fitness function that finds the optimal solution to solve a problem by iteratively enhancing the candidate solution. The optimized weights are processed using the TOPSIS algorithm that forms a decision matrix using the value of each criterion with each alternative. Furthermore, the decision matrix is now normalized and multiplied with the criteria weights. Distance measures are calculated between the positive-ideal and negative-ideal solutions [24]. Based on the relative closeness to the ideal solution, the alternatives are ranked, and this ranking provides a decision regarding the best location for the testing center.

The proposed work is organized as follows: Section 2 discusses in detail the existing work.  Section 3 explains the methodology of the proposed system.  Section 4 explains numerical examples in detail, and Section 5 provides the conclusion and future work of the proposed system.

## 2. Related Works

Social distancing is the best fighting strategy against COVID-19, which imposed lockdown throughout the world. There is a large dent in the economy worldwide as all the nonessential services are forced to close. The COVID-19 pandemic has prompted many researchers throughout the world to develop medicines, vaccines, and other treatment strategies that can help patients and healthcare workers. A careful strategy for efficient diagnosis is needed immediately as the number of confirmed cases is increasing hugely. The proposed work helps the government in determining the best location of the testing center for COVID-19.

The traditional strength weakness opportunity threat (SWOT) analysis is frequently used to assist decision-makers in qualitatively evaluating their competitiveness [25]. By dealing with statistical data, quantitative SWOT analysis methods such as competitive profile matrix (CPM), internal factor evaluation matrix (IFE), external factor evaluation matrix (EFE), and others differ from traditional SWOT analysis [26]. These methods have the disadvantage of not being able to examine both qualitative and quantitative data at the same time. The association between the COVID-19 testing center sites throughout the states of India is evaluated using fuzzy AHP, which assesses both qualitative and quantitative criteria at the same time.

Chou et al. [27] suggested a new fuzzy multiple-attribute decision-making (MADM) method for solving the facility location selection problem that uses objective and subjective criteria. In the Pacific Asian region, Lee and Lin [28] created a fuzzy quantitative SWOT analysis method for evaluating the competitive environment of international distribution hubs. To cope with quantitative and qualitative parameters in the location selection process, a fuzzy MCDM technique was presented in [29–32].

Li et al. [33] created a TOPSIS model for determining the site of a logistics center based on five criteria: traffic, communication, candidate land area, candidate land value, and freight transportation. Nanmaran et al. [34] proposed a model that combined the analytic network process (ANP), TOPSIS, and DEMATEL approaches to determine the location of an international distribution center based on criteria such as location resistance, extension transportation, port rate, one-stop service, import and export volume, convenience, transshipment time, port operation system, information abilities, and port and warehouse facilitation. Using this method, decision-makers cannot select candidate locations at the same time [35–37]. An evaluation model is developed for TQM consultant selection [38] that combined fuzzy TOPSIS with GP. The TOPSIS technique is applied to solve various MCDM problems such as multiprocessor scheduling [39], transformer oil grading [40, 41], transshipment site location selection [42], facility location selection [43], plant location selection [44], logistic center location selection [45], and evolutionary algorithm ranking [46] in different fields for the purpose of ranking and selection. But it demands the user to feed the weights associated with the different criteria. In the presented work, this problem is eradicated by employing fuzzy AHP for weight generation and a monkey search algorithm for weight optimization. The fuzzy clustering method is applied to control the spread of the virus in [47]. In [48], Multi-Criteria Decision Analysis is used to rank the hospital admissions of COVID-19 patients. These three works motivated the authors to apply the blend of three techniques to the testing center location selection problem. The proposed effort adds to the current research as well as has practical relevance. This paper shows how to combine MCDM techniques with metaheuristic methodologies for the decision-making problem. The comprehensive analysis of this study supplemented previous research by identifying a set of five essential characteristics to consider when deciding where to conduct the testing.

## 3. Methodology

The proposed work is aimed at finding the best location for the COVID-19 testing center that benefits the affected individual. The criteria considered are area, population, number of existing testing centers, patient density, and death rate. The alternatives assumed are 37 districts situated in Tamil Nadu. Fuzzy AHP (analytic hierarchy process) is deployed to compute weights of the decision criteria. Fuzzy AHP is one of the best methodologies for multiple criteria decision-making (MCDM) problems. It solves the problem by using triangular fuzzy numbers for pairwise comparison of various alternatives with different criteria and provides a decision for the MCDM problem.

A three-stage process has been applied for the selection of best locations for COVID-19 testing centers (Figure 1). The three stages of the research methodology are described in the following subsections.

### 3.1. Stage 1: Fuzzy AHP

The analytic hierarchy process (AHP) is a technique introduced by Saaty [49] for computing the weights of the involved decision criteria. The triangular fuzzy numbers and their corresponding linguistic terms as suggested by Saaty [49] are given in Table 1. In the decision-making process, AHP considers both qualitative and quantitative elements. AHP uses a discrete scale of 1 to 9 to decide the priorities of different attributes. Since the basic AHP does not deal with the uncertainty, vagueness, and ambiguity present in personal judgements, the proposed work applies the fuzzy AHP method to compute weights of the decision criteria. The supply chain vendor selection problem [50], the dry port location selection challenge in China [51], the thermal power plant location selection problem [52], the solar power plant location selection problem [53], and the wind power plant location selection problem [54] have all recently been solved by utilizing the fuzzy AHP method. Recently, some researchers have utilized neutrosophic functions for applications like scheduling [55–58] and for security enhancement [59–66]. Pairwise comparisons in fuzzy AHP are made using linguistic variables, which are represented as triangular numbers.

The different steps involved in fuzzy AHP are as follows:

**Step 1 (pairwise comparison matrix construction (D)).**

The construction of the pairwise comparison matrix involves the comparison of different criteria (area, population, number of affected patients, number of active patients, and number of deaths) involved in the location selection process with one another using Table 1.

When comparing the criteria of area and population, for example, if we believe that area is marginally more essential than population, the triangular fuzzy number is used (2,3,4). It also takes the value of (1/4, 1/3, 1/2) when comparing the population to the area. All of the remaining criteria are compared in the same way, and the pairwise comparison matrix is filled.

(1) $$\begin{array}{c} D=\left[\begin{array}{ccc} {\overset{ˇ}{d}}_{11} & \cdots & {\overset{ˇ}{d}}_{15}\\ \vdots & \ddots & \vdots \\ {\overset{ˇ}{d}}_{51} & \cdots & {\overset{ˇ}{d}}_{55} \end{array}\right]. \end{array}$$

**Step 2 (geometric mean calculation $\left({\overset{ˇ}{r}}_{i}\right)$).**

Geometric mean is calculated for each criterion using the following equation.

(2) $$\begin{array}{c} {\overset{ˇ}{r}}_{i}={\left(\overset{5}{\underset{j=1}{\prod }}{\overset{ˇ}{d}}_{ij}\right)}^{1/5},i=1,2,\cdots ,5. \end{array}$$

Next, the total geometric mean is calculated by summing up all geometric means.

**Step 3 (fuzzy weight calculation $\left({\overset{ˇ}{w}}_{i}\right)$).**

Relative fuzzy weights are calculated for each criterion using the following equation and (*lw*_*i*,_*mw*_*i*_, *uw*_*i*_) are triangular fuzzy numbers.

(3) $$\begin{array}{c} {\overset{ˇ}{w}}_{i}={\overset{ˇ}{r}}_{i}⊗{\left({\overset{ˇ}{r}}_{1}⊕{\overset{ˇ}{r}}_{2}⊕\cdots {\overset{ˇ}{r}}_{n}\right)}^{-1}, \end{array}$$

(4) $$\begin{array}{c} {\overset{ˇ}{w}}_{i}=\left({lw}_{i,}{mw}_{i},{uw}_{i}\right). \end{array}$$

**Step 4 (defuzzification of fuzzy weights (W_*i*_)).**

Fuzzy weights ${\overset{ˇ}{w}}_{i}$ need to be converted into a crisp number **W**_**i**_ by following the center of area method.

(5) $$\begin{array}{c} W_{i}=\frac{{lw}_{i}+{mw}_{i}+{uw}_{i}}{3}. \end{array}$$

**Step 5 (normalization of weights (NW_i_)).**

Calculate crisp weights are normalized using the following equation.

(6) $$\begin{array}{c} NW_{i}=\frac{W_{i}}{\sum_{i=1}^{n}W_{i}}. \end{array}$$

### 3.2. Stage 2: Monkey Search Algorithm

The monkey search algorithm (MSA) is a recently created metaheuristic algorithm that is based on a simulation of a monkey's mountain climbing procedure. The size of the monkey population is initially determined in MSA. The monkey's positions are then created at random between 0 and 1. The monkeys' position is then altered as a result of the step-by-step climbing procedure. Each monkey reaches the peak of their mountain after completing the climb. If a higher peak is discovered, the monkey will leap, relying on its eyesight. A monkey's eyesight is defined as the maximum distance at which they can watch. The position will be updated. The monkeys then use the present places as a pivot to find new searching domains. The monkeys will be in a different posture after this stage, which is known as the somersault process. If the number of iterations is reached, the procedure will be terminated. The following lists the drawbacks of using the traditional techniques (AHP and TOPSIS).

- Interdependency between criteria and alternatives
- Inconsistencies between judgment and ranking criteria
- Rank reversal
- No consideration of the correlation of attributes by the Euclidean distance
- Difficulty in keeping consistency of judgment

To overcome the limitations and to reap the following benefits, metaheuristic techniques like monkey search algorithm (MSA) are added to the traditional techniques (AHP and TOPSIS).

- Optimal weights
- Algorithm specific parameters (not required)
- The number of iterations
- Fitness evaluation

The somersault process of MSA makes monkeys find new search domains, and this avoids running into local search. Due to this, MSA is preferred in the proposed work when compared to other metaheuristic techniques, and the flowchart is given in Figure 2.

**Step 6 (solution representation and initialization).**

This step defines the population size of monkeys (M), and its position **x**_**i**_ = (**x**_**i**1_, **x**_**i**2_, ⋯, **x**_in_) of the optimization problem with *n* dimensions. The proposed work generates one solution from fuzzy AHP, and the remaining solutions are random solutions. Initialization of the population has a significant impact on precision in metaheuristic approaches. The initial populations of possible solutions in the original MSA are generated at random. If the solutions are initialized to very high or very low values in random initialization, a significant number of iterations are required to acquire the optimum weights. Hence, the proposed work uses one solution from fuzzy AHP and four random initial solutions.

**Step 7 (climb process).**

In this step, the position of the monkey is updated by considering the velocities of the monkeys.

For the first iteration, use the velocity as, **v**_**ij**_^0^ = *v*_min_ + (*v*_max_ − *v*_min_)∗*r*_2_, where *v*_min_ = −4.0 and *v*_max_ = 4.0, then for the next consecutive iteration use, **v**_**ij**_^**t**^ = **w**^**t**−1^**v**^**t**−1^ + *c*_1_*r*_1_(**p**_**ij**_^**t**−1^ − **x**_**ij**_^**t**−1^) + *c*_2_*r*_2_(**g**_**j**_^**t**−1^ − **x**_**ij**_^**t**−1^).

*c*_1_ and *c*_2_ are acceleration coefficients, and they are assigned the value of 2; *r*_1_ and *r*_2_ are random numbers assigned between (0,1), **g**_**j**_ is the global best, **p**_**ij**_ is the personal best, **w** is the inertia weight, and initially, it is set to *w*^0^ = 0.9, and it is updated in the successive iterations using, **w**^**t**^ = **w**^**t**−1^∗df, where df is the decrement factor, and it is taken as 0.975, and the position of the monkeys is updated using **x**_**new**_ = **x**_**old**_ + **v**.

**Step 8 (swap process).**

This step selects two monkeys randomly and swaps their positions to improve the current solution.

**Step 9 (watch-jump process).**

This step updates the position of the monkeys by randomly generating a real number (*y*) in the interval (**x**_**ij**_–**b**, **x**_**ij**_ + *b*), where “*b*” is the eyesight of the monkey, which indicates the maximum distance that the monkey could watch. If **f**(**x**) < **f**(**y**), then update **x** with the newly generated number else repeat the process.

**Step 10 (somersault process).**

This step updates the position of the monkeys by randomly generating a real number “*z*” from the somersault interval [*c*, *d*] = [−1, 1].  **y**_**i**_ = **x**_**ij**_ + *z*(**p**_**j**_ − **x**_**ij**_). If **f**(**x**) < **f**(**y**), then update *x* with the newly generated number else repeat the process.

Where *p* is the somersault pivot, **p**_**j**_ = (1/**M**)∑_**i**=1_^**M**^**x**_**ij**_.

**Step 11 (termination).**

The above steps are repeated until the stopping criterion is met. The number of iterations (200) is used as a stopping criterion in this work.

### 3.3. Stage 3: TOPSIS

TOPSIS is a common multicriteria decision-making process that ranks and orders options based on their distance from the positive and negative ideal solutions. This method considers an option to be the greatest if it is the closest to a positive ideal solution and the furthest away from a negative ideal solution. The positive ideal solution is the one that has the highest value for all of the criteria that have been considered. The negative ideal solution is the one that has the lowest value for all of the criteria taken into account.

Let **C**^+^ represent the set of benefit criteria (the higher the number, the better) and **C**^−^represent the set of cost criteria (the lower the number, the better) (less is better). The TOPSIS approach involves the following steps:

**Step 12 (construction of performance score matrix (*X*)_*m*×*n*_).**

Create a performance score matrix (*X*)_*m*×*n*_ consisting of *m* alternatives and *n* criteria, by filling the intersection of each alternative and criteria with the evaluation value given as *X*_**ij**_.

**Step 13 (construction of normalized decision matrix (N_ij_)).**

Because the performance values of alternatives for different criteria will have different dimensions, this step is required. To have a uniform effect and to allow comparisons across criteria, the performance score matrix is normalized.

(7) $$\begin{array}{c} N_{ij}=\frac{X_{ij}}{\sqrt{\sum_{i=1}^{m}X_{ij}^{2}}},i=1,2,\cdots ,m\text{ and }j=1,2,\cdots ,n. \end{array}$$

**Step 14 (construction of weighted normalized decision matrix (V_ij_)).**

This step uses the optimized weight vector (**w**_**j**_) generated in the previous stage. It entails multiplying each column of the normalized decision matrix by the weight assigned to it. The following formula is used to calculate the weighted normalized decision matrix:

(8) $$\begin{array}{c} V_{ij}=w_{j}*N_{ij}. \end{array}$$

**Step 15 (identification of positive and negative ideal solution (V^+^and V^−^)).**

The following equations can be used to find the positive ideal solution and the negative ideal solution:

(9) $$\begin{array}{c} V^{+}=\left\{\left(\max\;V_{ij}\left|\;j=C^{+}\right.\right),\left(\min\;V_{ij}\left|j=C^{-}\right.\right)\right\}\forall i=1,2,..,m, \end{array}$$

(10) $$\begin{array}{c} V^{+}=\left\{V_{1}^{+},V_{2}^{+},\cdots ,V_{m}^{+}\right\}, \end{array}$$

(11) $$\begin{array}{c} V^{-}=\left\{\left(\min\;V_{ij}\left|\;j=C^{+}\right.\right),\left(\max\;V_{ij}\left|j=C^{-}\right.\right)\right\}\forall i=1,2,\cdots ,m, \end{array}$$

(12) $$\begin{array}{c} V^{-}=\left\{V_{1}^{-},V_{2}^{-},\cdots ,V_{m}^{-}\right\}. \end{array}$$

**Step 16 (calculation of separation measure (S_i_^+^and S_i_^−^)).**

In this phase, the separation measure of an alternative from the positive ideal solution and the negative ideal solution is calculated. The following formula is used to determine the separation measure from a positive ideal solution:

(13) $$\begin{array}{c} S_{i}^{+}=\sqrt{\overset{j=n}{\underset{j=1}{\sum }}{\left(V_{j}^{+}-V_{ij}\right)}^{2}\forall }i=1,2,\cdots ,m. \end{array}$$

Separation measure from negative ideal solution is calculated as follows:

(14) $$\begin{array}{c} S_{i}^{-}=\sqrt{\overset{j=n}{\underset{j=1}{\sum }}{\left(V_{j}^{-}-V_{ij}\right)}^{2}\forall }i=1,2,\cdots ,m. \end{array}$$

**Step 17 (relative closeness coefficient calculation (RC_i_^∗^)).**

This stage compares the alternatives by taking into account both the positive and negative ideal solutions. The value of the relative closeness coefficient is computed as follows:

(15) $$\begin{array}{c} {RC}_{i}^{*}=\frac{S_{i}^{-}}{\left(S_{i}^{+}+S_{i}^{-}\right)}. \end{array}$$

Choose the alternative with a high relative closeness coefficient **RC**_**i**_^∗^ value. The alternatives are assigned ranks based on the relative closeness coefficient **RC**_**i**_^∗^ value in decreasing order.

## 4. Numerical Example

This section uses a numerical example to demonstrate the applicability of the proposed method. The Java programming language was used to implement all of the steps.

### 4.1. Stage 1: Fuzzy AHP

**Step 18 (pairwise comparison matrix).**

A 5 × 5 pairwise comparison matrix is constructed as the proposed work deals with five criteria. The matrix is filled with triangular fuzzy numbers according to their relative importance, as shown in Table 2.

**Step 19 (geometric mean).**

This step uses equation (2) to find the geometric mean of each criterion, and the result is shown in Table 3.

**Step 20 (relative fuzzy weight of each criterion).**

This step uses equations (3) and (4) to calculate the relative fuzzy weight of each criterion, which is shown in Table 4.

**Step 21 (crisp weight of each criterion).**

This step calculates the crisp weight of each criterion by defuzzifying the fuzzy weights created in the previous step using the center of area method discussed in equation (5), and it is given in Table 5.

**Step 22 (normalized weight of each criterion).**

Crisp weights are normalized using equation (6), and it is given in Table 6.

### 4.2. Stage 2: MSA

**Step 23 (solution representation and initialization).**

This step initializes the initial population as given in Table 7, population size (=5) and other algorithm-specific parameters.

**Step 24 (climb process).**

The position of the monkey is updated using the monkeys' velocities in this stage, as shown in Table 8.

**Step 25 (swap process).**

This step selects two monkeys randomly and swaps their positions to improve the current solution. It is given in Table 9.

**Step 26 (watch-jump process).**

This step updates the position of the monkeys using eyesight, and the result is given in Table 10.

**Step 27 (somersault process).**

This step updates the position of the monkeys by randomly generating a real number “*z*” from the somersault interval, and it is given in Table 11.

Then, Steps 2, 3, 4, and 5 are carried out for 200 iterations as illustrated in Figure 3, and then, the best solution is found as given below: *x*_1_ = 0.081, *x*_2_ = 0.172, *x*_3_ = 0.031, *x*_4_ = 0.312, and *x*_5_ = 0.404.

### 4.3. Stage 3: TOPSIS

**Step 28 (construction of performance score matrix).**

The performance score of alternatives against the various criteria as on August 7, 2020, is given in Table 12.

**Step 29 (construction of normalized decision matrix).**

The normalized decision matrix is constructed from the performance score matrix by using equation (7), and it is shown in Table 13.

**Step 30 (construction of weighted normalized decision matrix).**

The weighted normalized decision matrix is constructed from the normalized decision matrix using equation (8), and it is given in Table 14.

**Step 31 (identification of positive and negative ideal solution).**

Positive and negative ideal solutions are obtained by using equations (10) and (12), respectively, and they are shown in Table 15.

**Step 32 (calculation of separation measure).**

Separation measures are calculated for each alternative from positive and negative ideal solutions using equations (13) and (14), respectively, and it is shown in Table 16.

**Step 33 s 6 and 7 (relative closeness coefficient and rank calculation).**

Relative closeness coefficient values for the alternatives are computed using equation (15). According to the relative closeness coefficient value, the alternatives are assigned a rank (the higher the score, the least rank is assigned) and given in Table 17.

The proposed technique has given the top three COVID-19 testing center locations as Chennai, followed by Chengalpet, and then Thiruvallur.

As it is inferred from the data, in the number of affected patients, Chennai stood first. To reflect this situation, our proposed system has assigned rank 1 to the Chennai district, followed by Chengalpet and then Thiruvallur. Similarly, the last few ranks are assigned to Ariyalur, Perambalur, and Udagamandalam, where the severity of the disease is relatively less when compared to other districts.

## 5. Conclusion

In this paper, we proposed a combination of three approaches, namely, fuzzy AHP, MSA, and TOPSIS, for the choice of COVID-19 testing center location for any state. The COVID-19 testing labs play a vital role in controlling the spread of novel coronavirus. The leading medical professionals and government officials are investing time and energy in the location selection procedure, since inappropriate location selection might bring about loss and affect many human lives. This paper proposed a novice solution using a blend of three approaches to solve the location selection problem. For optimizing the weights generated by fuzzy AHP, MSA is chosen. Moreover, TOPSIS stands at the first position in the ranking/selection procedure to help the officials decide the location for a particular state. The main limitation of the proposed work is that if the pairwise comparison matrix is not properly constructed in the fuzzy AHP stage, it will affect the subsequent steps. This, in turn, will have a great impact on ranking results. Hence, there is a need to have a greater emphasis on the pairwise comparison matrix construction. To effectively optimize the weights, future works of interest could replace MSA with other metaheuristic algorithms. In addition to this problem, the proposed solution can be applied to various fields, such as institution/faculty selection in the educational domain and hospital/doctor selection in the healthcare domain.

## Figures and Tables

**Figure 1:** Overview of the proposed work.

**Figure 2:** Flowchart of monkey search algorithm.

**Figure 3:** Number of iterations versus fitness function in MSA.

**Table 1:** Saaty scale and its equivalent triangular fuzzy number.

Saaty scale	Linguistic terms	Triangular fuzzy number
1	Equally important	(1,1,1)
3	Weakly important	(2,3,4)
5	Fairly important	(4,5,6)
7	Strongly important	(6,7,8)
9	Absolutely important	(9,9,9)

**Table 2:** Pairwise comparison matrix.

Criteria	Area			Population			No. of affected patients			No. of active patients			Death		
Area	1	1	1	1/4	1/3	1/2	2	3	4	1/4	1/3	1/2	1/4	1/3	1/2
Population	2	3	4	1	1	1	2	3	4	1/4	1/3	1/2	1/4	1/3	1/2
No. of affected patients	1/4	1/3	1/2	1/4	1/3	1/2	1	1	1	1/6	1/5	1/4	1/4	1/3	1/2
No. of active patients	2	3	4	2	3	4	4	5	6	1	1	1	1	1	1
Death	2	3	4	2	3	4	2	3	4	1	1	1	1	1	1

**Table 3:** Geometric mean of criteria.

Criteria	${\overset{ˇ}{r}}_{i}$		
Area	0.500	0.644	0.871
Population	0.758	1.000	1.320
No. of affected patients	0.304	0.375	0.500
No. of active patients	1.741	2.141	2.491
Death	1.516	1.933	2.297
Total	4.819	6.094	7.479

**Table 4:** Fuzzy weight of criteria.

Criteria	${\overset{ˇ}{w}}_{i}$		
Area	0.067	0.106	0.181
Population	0.101	0.164	0.274
No. of affected patients	0.041	0.062	0.104
No. of active patients	0.233	0.351	0.517
Death	0.203	0.317	0.477

**Table 5:** Crisp weight of criteria.

Criteria	*W*_*i*_
Area	0.118
Population	0.180
No. of affected patients	0.069
No. of active patients	0.367
Death	0.332

**Table 6:** Normalized weight of criteria.

Criteria	NW_*i*_
Area	0.111
Population	0.169
No. of affected patients	0.064
No. of active patients	0.345
Death	0.312
Total	1.000

**Table 7:** Initial population.

Monkeys	*x*_1_	*x*_2_	*x*_3_	*x*_4_	*x*_5_
1	0.111	0.169	0.064	0.345	0.312
2	0.134	0.255	0.452	0.101	0.058
3	0.374	0.121	0.258	0.072	0.175
4	0.235	0.262	0.092	0.287	0.124
5	0.325	0.111	0.189	0.132	0.243

**Table 8:** Population after climb process.

Monkeys	*x*_1_	*x*_2_	*x*_3_	*x*_4_	*x*_5_
1	0.095	0.153	0.069	0.372	0.311
2	0.165	0.234	0.442	0.112	0.047
3	0.333	0.149	0.264	0.09	0.164
4	0.265	0.287	0.105	0.217	0.126
5	0.325	0.118	0.196	0.125	0.236

**Table 9:** Population after swap process.

Monkeys	*x*_1_	*x*_2_	*x*_3_	*x*_4_	*x*_5_
1	0.095	0.153	0.069	0.372	0.311
2	0.165	0.234	0.442	0.112	0.047
3	0.325	0.118	0.196	0.125	0.236
4	0.265	0.287	0.105	0.217	0.126
5	0.333	0.149	0.264	0.09	0.164

**Table 10:** Population after watch-jump process.

Monkeys	*x*_1_	*x*_2_	*x*_3_	*x*_4_	*x*_5_
1	0.095	0.138	0.069	0.388	0.31
2	0.165	0.234	0.442	0.112	0.047
3	0.325	0.118	0.196	0.125	0.236
4	0.265	0.287	0.105	0.217	0.126
5	0.369	0.149	0.221	0.097	0.164

**Table 11:** Population after somersault process.

Monkeys	*x*_1_	*x*_2_	*x*_3_	*x*_4_	*x*_5_
1	0.092	0.112	0.064	0.386	0.346
2	0.165	0.234	0.442	0.112	0.047
3	0.3	0.147	0.196	0.119	0.238
4	0.265	0.287	0.105	0.217	0.126
5	0.369	0.149	0.221	0.097	0.164

**Table 12:** Performance score matrix.

Alternatives	Area	Population	No. of affected patients	No. of active patients	Death
Ariyalur	1940	754894	1154	218	10
Chengalpet	2944.46	2556244	16897	2644	284
Chennai	178.2	4646732	106096	11720	2248
Coimbatore	4723	3458045	5997	1579	96
Cuddalore	3678	2605914	4232	1912	49
Dharmapuri	4497.77	1506843	815	86	7
Dindigul	6266.64	2159775	3331	561	63
Erode	8161.91	2251744	888	239	13
Kallakurichi	3520.37	1370281	4131	827	30
Kanchipuram	1655.94	1166401	10993	2872	137
Karur	2895.57	1064493	680	319	10
Krishnagiri	5143	1883731	1263	449	16
Madurai	3741.73	3038252	11689	1864	276
Nagapattinam	2715.83	1616450	921	390	11
Kanyakumari	1672	1870374	5829	1933	63
Namakkal	3368.21	1726601	890	363	10
Perambalur	1757	565223	572	142	9
Pudukottai	4663	1618345	2755	821	33
Ramanathapuram	4068.31	1353445	3503	389	71
Ranipet	2234.32	1210277	6342	1731	44
Salem	5205	3482056	4251	1109	43
Sivagangai	4086	1339101	2768	460	55
Tenkasi	2916.13	1407627	2629	870	39
Thanjavur	3396.57	2405890	3484	881	36
Theni	3066	1245899	6836	2686	82
Thiruvallur	3422.23	3728104	15890	3469	268
Thiruvarur	2161	1264277	1874	181	12
Thoothukudi	4621	1750176	8450	1832	61
Tiruchirappalli	4407	2722290	4834	1273	67
Tirunelveli	3842.37	1665253	6071	2274	65
Tirupattur	1792.92	1111812	1436	489	25
Tiruppur	5186.34	2479052	1059	329	18
Tiruvannamalai	6191	2464875	7058	1995	81
Udagamandalam	2452.5	735394	919	160	3
Vellore	2080.11	1614242	6897	1376	81
Viluppuram	3725.54	2093003	4316	803	40
Virudhunagar	4288	1942288	9441	1911	114

**Table 13:** Normalized decision matrix.

Alternatives	Area	Population	No. of affected patients	No. of active patients	Death
Ariyalur	0.081799328	0.058125508	0.010252	0.014887	0.004309
Chengalpet	0.124151984	0.196826286	0.150111	0.180553	0.122372
Chennai	0.007513732	0.35779018	0.942543	0.800333	0.968633
Coimbatore	0.199143415	0.266263374	0.053277	0.107826	0.041365
Cuddalore	0.155081406	0.200650788	0.037597	0.130566	0.021113
Dharmapuri	0.189646682	0.116024257	0.00724	0.005873	0.003016
Dindigul	0.264230381	0.166298871	0.029592	0.038309	0.027146
Erode	0.344143686	0.173380322	0.007889	0.016321	0.005602
Kallakurichi	0.148435	0.105509224	0.036699	0.056474	0.012927
Kanchipuram	0.069822051	0.089810823	0.09766	0.196122	0.059031
Karur	0.122090556	0.081964086	0.006041	0.021784	0.004309
Krishnagiri	0.216852548	0.145043969	0.01122	0.030661	0.006894
Madurai	0.157768556	0.233940053	0.103843	0.127288	0.118925
Nagapattinam	0.114511891	0.124463803	0.008182	0.026632	0.00474
Kanyakumari	0.070499214	0.144015504	0.051784	0.132	0.027146
Namakkal	0.142019234	0.132945236	0.007907	0.024788	0.004309
Perambalur	0.074083206	0.043521175	0.005082	0.009697	0.003878
Pudukottai	0.196613539	0.124609715	0.024475	0.056064	0.014219
Ramanathapuram	0.171538672	0.104212881	0.03112	0.026564	0.030593
Ranipet	0.094209213	0.093189197	0.056341	0.118206	0.018959
Salem	0.219466753	0.268112179	0.037765	0.075731	0.018528
Sivagangai	0.172284564	0.103108418	0.024591	0.031412	0.023699
Tenkasi	0.122957461	0.1083848	0.023356	0.05941	0.016805
Thanjavur	0.143215022	0.185249293	0.030951	0.060162	0.015512
Theni	0.12927667	0.095932029	0.06073	0.183421	0.035333
Thiruvallur	0.144296966	0.287057442	0.141165	0.23689	0.115478
Thiruvarur	0.091117705	0.097347102	0.016648	0.01236	0.005171
Thoothukudi	0.194842626	0.134760469	0.075069	0.125103	0.026284
Tiruchirappalli	0.185819401	0.209611535	0.042945	0.08693	0.028869
Tirunelveli	0.162012002	0.128221548	0.053934	0.155286	0.028008
Tirupattur	0.075597758	0.085607566	0.012757	0.033393	0.010772
Tiruppur	0.218679962	0.190882638	0.009408	0.022467	0.007756
Tiruvannamalai	0.261041051	0.189791034	0.062702	0.136234	0.034902
Udagamandalam	0.103408686	0.056624043	0.008164	0.010926	0.001293
Vellore	0.08770701	0.124293791	0.061272	0.093964	0.034902
Viluppuram	0.157085911	0.161157545	0.038343	0.054835	0.017235
Virudhunagar	0.180801813	0.149552755	0.083873	0.130498	0.049121

**Table 14:** Weighted normalized decision matrix.

Alternatives	Area	Population	No. of affected patients	No. of active patients	Death
Ariyalur	0.006625746	0.009997587	0.000318	0.004645	0.001741
Chengalpet	0.010056311	0.033854121	0.004653	0.056332	0.049438
Chennai	0.000608612	0.061539911	0.029219	0.249704	0.391328
Coimbatore	0.016130617	0.0457973	0.001652	0.033642	0.016712
Cuddalore	0.012561594	0.034511936	0.001165	0.040737	0.00853
Dharmapuri	0.015361381	0.019956172	0.000224	0.001832	0.001219
Dindigul	0.021402661	0.028603406	0.000917	0.011953	0.010967
Erode	0.027875639	0.029821415	0.000245	0.005092	0.002263
Kallakurichi	0.012023235	0.018147586	0.001138	0.01762	0.005222
Kanchipuram	0.005655586	0.015447461	0.003027	0.06119	0.023849
Karur	0.009889335	0.014097823	0.000187	0.006797	0.001741
Krishnagiri	0.017565056	0.024947563	0.000348	0.009566	0.002785
Madurai	0.012779253	0.040237689	0.003219	0.039714	0.048046
Nagapattinam	0.009275463	0.021407774	0.000254	0.008309	0.001915
Kanyakumari	0.005710436	0.024770667	0.001605	0.041184	0.010967
Namakkal	0.011503558	0.022866581	0.000245	0.007734	0.001741
Perambalur	0.00600074	0.007485642	0.000158	0.003025	0.001567
Pudukottai	0.015925697	0.021432871	0.000759	0.017492	0.005745
Ramanathapuram	0.013894632	0.017924616	0.000965	0.008288	0.01236
Ranipet	0.007630946	0.016028542	0.001747	0.03688	0.007659
Salem	0.017776807	0.046115295	0.001171	0.023628	0.007485
Sivagangai	0.01395505	0.017734648	0.000762	0.009801	0.009574
Tenkasi	0.009959554	0.018642186	0.000724	0.018536	0.006789
Thanjavur	0.011600417	0.031862878	0.000959	0.01877	0.006267
Theni	0.01047141	0.016500309	0.001883	0.057227	0.014274
Thiruvallur	0.011688054	0.04937388	0.004376	0.07391	0.046653
Thiruvarur	0.007380534	0.016743702	0.000516	0.003856	0.002089
Thoothukudi	0.015782253	0.023178801	0.002327	0.039032	0.010619
Tiruchirappalli	0.015051371	0.036053184	0.001331	0.027122	0.011663
Tirunelveli	0.013122972	0.022054106	0.001672	0.048449	0.011315
Tirupattur	0.006123418	0.014724501	0.000395	0.010419	0.004352
Tiruppur	0.017713077	0.032831814	0.000292	0.00701	0.003133
Tiruvannamalai	0.021144325	0.032644058	0.001944	0.042505	0.0141
Udagamandalam	0.008376104	0.009739335	0.000253	0.003409	0.000522
Vellore	0.007104268	0.021378532	0.001899	0.029317	0.0141
Viluppuram	0.012723959	0.027719098	0.001189	0.017109	0.006963
Virudhunagar	0.014644947	0.025723074	0.0026	0.040715	0.019845

**Table 15:** Positive and negative ideal solution.

Positive and negative ideal solution	Area	Population	No. of affected patients	No. of active patients	Death
*V* ^+^	0.027875639	0.061539911	0.029219	0.249704	0.391328
*V* ^−^	0.000608612	0.007485642	0.000158	0.001832	0.000522

**Table 16:** Separation measure.

Alternatives	*S*_*i*_^+^	*S*_*i*_^−^
Ariyalur	0.464516	0.007207
Chengalpet	0.394928	0.078535
Chennai	0.027267	0.466836
Coimbatore	0.433781	0.054634
Cuddalore	0.438125	0.049517
Dharmapuri	0.465136	0.01933
Dindigul	0.450697	0.033022
Erode	0.461575	0.035441
Kallakurichi	0.453721	0.022722
Kanchipuram	0.416992	0.064534
Karur	0.462816	0.012489
Krishnagiri	0.45925	0.02564
Madurai	0.404099	0.070169
Nagapattinam	0.461204	0.017687
Kanyakumari	0.436761	0.044548
Namakkal	0.461444	0.019789
Perambalur	0.465842	0.00562
Pudukottai	0.452944	0.026495
Ramanathapuram	0.452542	0.021632
Ranipet	0.442415	0.037472
Salem	0.446735	0.048079
Sivagangai	0.454105	0.020712
Tenkasi	0.451975	0.023033
Thanjavur	0.451161	0.032181
Theni	0.42696	0.058645
Thiruvallur	0.388241	0.096012
Thiruvarur	0.463895	0.011758
Thoothukudi	0.437793	0.044351
Tiruchirappalli	0.441904	0.042306
Tirunelveli	0.432953	0.051583
Tirupattur	0.458806	0.013087
Tiruppur	0.459739	0.031123
Tiruvannamalai	0.432268	0.053819
Udagamandalam	0.466147	0.008241
Vellore	0.44007	0.034322
Viluppuram	0.451659	0.028846
Virudhunagar	0.428768	0.049202

**Table 17:** Relative closeness coefficient and rank.

Alternatives	RC_*i*_^∗^	Rank
Ariyalur	0.015277	36
Chengalpet	0.165874	3
Chennai	0.944815	1
Coimbatore	0.11186	7
Cuddalore	0.101545	11
Dharmapuri	0.039899	30
Dindigul	0.068267	19
Erode	0.071307	18
Kallakurichi	0.04769	26
Kanchipuram	0.134019	5
Karur	0.026276	33
Krishnagiri	0.052878	24
Madurai	0.147952	4
Nagapattinam	0.036934	31
Kanyakumari	0.092556	13
Namakkal	0.041121	29
Perambalur	0.011921	37
Pudukottai	0.055263	23
Ramanathapuram	0.04562	27
Ranipet	0.078084	16
Salem	0.097165	12
Sivagangai	0.04362	28
Tenkasi	0.04849	25
Thanjavur	0.06658	20
Theni	0.120767	6
Thiruvallur	0.198269	2
Thiruvarur	0.02472	34
Thoothukudi	0.091987	14
Tiruchirappalli	0.087371	15
Tirunelveli	0.106458	9
Tirupattur	0.027732	32
Tiruppur	0.063405	21
Tiruvannamalai	0.110719	8
Udagamandalam (Ootacamund)	0.017371	35
Vellore	0.072349	17
Viluppuram	0.060032	22
Virudhunagar	0.10294	10

## Data Availability

The data used to support the findings of this study are included in the article.
